# The Function and Prognostic Value of RNA-Binding Proteins in Colorectal Adenocarcinoma Were Analyzed Based on Bioinformatics of Smart Medical Big Data

**DOI:** 10.1155/2021/5536330

**Published:** 2021-06-02

**Authors:** Haoran Zhao, Peng Wang, Haishi Liu, Yueyang Li, Qian Luo, Man Li, Yubao Zhang, Zengfu Song

**Affiliations:** ^1^Department of Hepatopancreatobiliary Surgery, Harbin Medical University Cancer Hospital, Harbin, China; ^2^Key Laboratory of Hepatosplenic Surgery, Ministry of Education, Harbin Medical University, Harbin, China

## Abstract

Colon cancer is the third most frequent cancer in the world and is mainly adenocarcinoma in terms of pathological type. It has been confirmed that the dysregulation of RNA-binding proteins (RBPs) significantly participates in the occurrence and development of numerous malignant tumors. Therefore, we analyzed the RBPs associated with colon adenocarcinoma (COAD) to assess their possible biological effects and prognostic value. A total of 398 COAD tissue datasets and 39 normal tissue datasets were retrieved from the TCGA data resource and screened out the RBPs, which are differentially expressed between tumor tissues and nontumor tissues. Then, bioinformatics analyses based on smart medical big data were conducted on these RBPs. Overall, 181 differentially expressed RBPs were uncovered, consisting of 121 upregulated RBPs and 60 downregulated RBPs. Finally, we selected 7 prognostic-related RBPs with research prospects and constructed a prognostic model according to the median risk score. There were remarkable differences in OS between the high-risk and low-risk groups. In addition, the performance of the prognostic model was evaluated and verified with other COAD patient data in the TCGA database. The results showed that the area under the ROC curve (AUC) for the train group was 0.744 and the one for the test group was 0.661, confirming that the model assesses patients' prognosis to some extent. And based on 7 hub RBPs, we constructed a nomogram as a reference for evaluating the survival rate of COAD patients.

## 1. Introduction

Colorectal carcinoma is one of the most common gastrointestinal malignancies and the third most common cancer type in the world. Over 95% of colon cancer cases are adenocarcinoma in terms of pathology, and regions differ significantly in regard to epidemiological characteristics [1, 2]. The incidence of colon cancer is relatively high in western developed countries: taking the United States as an example, approximately 1,014,200 colon cancer patients are diagnosed each year [3]. Colon cancer tends to occur in middle-aged and elderly people. As the global population is expanding and aging, colon cancer is expected to cause 60% more deaths by 2035 [4]. The onset of colon cancer is relatively insidious, and most of the patients had no obvious early symptoms. So, patients often look for treatment after suffering from abdominal pain, gastrointestinal bleeding, and even metastasis [5, 6]. At present, colonoscopy is an effective method for screening colon cancer and removing precancerous lesions, which reduces the incidence and mortality of colon cancer [7]. However, since colonoscopy is an invasive test requiring inconvenient preparation, colon cleansing, and laboratory test, it is not widely accepted by the target population. Therefore, it is necessary to find an effective method for early screening, diagnosis, and prognosis evaluation based on the molecular mechanism of COAD.

RBPs refer to a group of proteins that can recognize the interaction between special RNA-binding domains and RNA, and they are significantly involved in the modulation of posttranscriptional gene expression. RBPs mainly work in regulating the stability of mRNA, splicing, editing and translation of RNA, mRNA localization, and polyadenylation [8]. There have been many reports on the mechanism of RBPs dysregulation affecting the key posttranscriptional steps involved in it. For example, RBP dysregulation makes it unable to combine with splicing factors to form DNA/RNA hybrids (R-loops), which play a key role in transcription and RNA processing, causing the RNA-induced genome less stable [9]. Upregulation of certain RBPs can affect their target mRNAs encode products; promote proliferation; inhibit apoptosis; and promote angiogenesis, cancer invasion, and metastasis [10]. At present, RBPs related to various malignant tumors have gradually attracted more attention and academic research [11–14]. Thus, the biological targets screened for the potential RBPs function have important significance for the diagnosis, treatment, and prognosis evaluation of the disease.

In recent years, the fact that the huge network of RBP and its target mRNA have worked in tumorigenesis and development has gradually attracted increasingly more attention. And the mechanism by which RBP affects the expression of many oncogenes has also been better understood. For instance, when the splicing factor SAM68 is overexpressed in cancer, which promotes the inclusion of exon v5 in the CD44 pre-mRNA and the generation of splicing factor SF2/ASF, deregulation of splicing and irregular protein expression occurs. This is how various types of malignant tumor develop [15–17]. The human antigen R (HuR) which is generally highly expressed in malignant tumors can stabilize the mRNAs encoding the cyclins (cyclin A2, B1, D1, and E1), participate transcripts encoding antiapoptotic factors (Bcl-2, Mcl-1, etc.), and encode the mRNA (MMP-9) that invades and transfer related protein. The above process will enhance proliferation, invasion along with metastasis of cancer cells [10]. The overexpression of Musashi RNA-binding protein (MSI), which is composed of two isozymes MSI1 and MSI2, will affect the regulation of mRNA stability and translation in various oncogenic signaling pathways (PTEN/mTOR, TGF*β*/SMAD3, cMET, etc.). Such overexpression promotes the invasion, development, and metastasis of cancer [18]. The above studies illustrate the correlation between RBPs and malignant tumors as well as RBPs' huge potential research value. Therefore, after analyzing COAD-related RBPs based on bioinformatics of smart medical big data, we screened out differentially expressed RBPs which are highly related to colorectal carcinoma and established a prognostic model, aiming to find some biomarkers that may be relevant for diagnosis along with prognosis.

## 2. Results

### 2.1. Identifying Differentially Expressed RBPs in Patients with COAD

Herein, we retrieved the dataset covering 398 COAD tissues and 39 nontumor tissues from the TCGA data repository and analyzed them based on the R language software package. Overall, 1543 RBPs were included, among which 181 RBPs were established as colon adenocarcinoma genes differentially expressed compared with normal samples. Setting the criteria of fold change greater than or equal to 1, as well as false discovery rate (FDR) less than 0.05, we targeted 121 upregulated RBPs and 60 downregulated RBPs (Figure 1).

### 2.2. GO and KEGG Enrichment Analysis of the Differently Expressed RBPs

We conducted GO categories along with KEGG pathways analyses on differentially expressed RBPs through R scripts. According to their expression, RBPs were defined as upregulated RBP and downregulated RBP. Covering three aspects, namely, molecular function (MF), biological process (BP), as well as cellular component (CC), the results of GO enrichment analysis revealed that, in the BP gone through GO enrichment analysis, the downregulated RBPs were primarily involved in the modulation of mRNA processing and metabolic process, RNA localization and phosphodiester bond hydrolysis, modulation of translation, modulation of cellular amide metabolic process, while the upregulated RBPs were enriched during ncRNA processing and metabolic process, nucleic acid phosphodiester bond hydrolysis, and the biogenesis of ribosome and ribonucleoprotein complex (Table 1). According to the cellular component (CC), the downregulated RBPs primarily participated in ribonucleoprotein granule, endolysosome, endolysosome membrane, and cytoplasmic ribonucleoprotein granule. However, the upregulated RBPs were abundant in the following steps: ribonucleoprotein granule, preribosome, cytoplasmic ribonucleoprotein granule, and P granule (Table 1). For the GO molecular function (MF), the downregulated RBPs were abundant in double-stranded RNA-binding, translation suppressor activity, mRNA 3′-UTR binding, and AU-rich element binding; the upregulated RBPs were mainly involved in catalytic activity acting on RNA, ribonuclease activity, nuclease activity, and mRNA 3′-UTR binding (Table 1). Moreover, based on the KEGG pathways analysis, the downregulated RBPs were largely associated with Oocyte meiosis, Toll-like receptor signaling cascade, and progesterone-mediated oocyte maturation, while the upregulated RBPs were associated with Ribosome biogenesis in eukaryotes mRNA surveillance cascade, and RNA transport, and degradation (Table 1).

### 2.3. Protein-Protein Interaction (PPI) Network Construction and Module Selection

Through the information of the STRING website, we evaluated the function of RBPs in COAD and created a PPI network that incorporated 150 nodes along with 574 edges, with the Cytoscape software. Then, we used the MCODE plugin in Cytoscape to screen key modules (38 nodes and 213 edges) from the coexpression network (Figure 2(a)). Genes in Module 1 mainly focused on RNA processing and metabolic process, preribosome catalytic activity acting on RNA, ribosome biogenesis, and ribonucleoprotein complex biogenesis (Figure 2(b)). And genes in Module 2 were primarily involved in RNA splicing, modulation of mRNA processing, and metabolic process (Figure 2(c)).

### 2.4. Selection and Verification of Prognosis-Related RBPs

We totally identified 135 key differently expressed RBPs from the PPI network and screened out 13 prognostic-linked candidate hub RBPs through univariate COX regression, including TERT, POP1, TDRD7, TDRD5, LUZP4, PPARGC1B, PPARGC1A, LIN28B, EIF4E3, LRRFIP2, RBM47, CELF4, and PNLDC1 (Figure 3). Subsequently, multivariate COX regression was carried out on these 13 candidate hub RBPs and spot 7 RBPs with the prospective potential prognosis ability, namely, POP1, TDRD7, TDRD5, PPARGC1A, LIN28B, LRRFIP2, and PNLDC1. Among them, TDRD5, LIN28B, and PNLDC1 (Figure 4), whose HR value was greater than 1, were demonstrated to risky prognostic genes, while POP1, TDRD7, PPARGC1A, and LRRFIP2, whose HR value was lower than 1, were found to be protective prognostic genes. After screening out RBPs related to prognosis, the expression of these RBPs of normal colon tissue and tumor tissue was validated by Human Protein Atlas (HPA): the levels of antibody staining of TDRD5 and LIN28B were significantly higher and the levels of antibody staining of PNLDC1, TDRD7, and LRRFIP2 were significantly weaker (Figure 5).

### 2.5. Construction and Analysis of Prognostic Model

Based on the above 7 selected hub RBPs, a prognostic model was built as follows:

Risk score = (−0.8328^∗^ExpPOP1) + (−1.6761^∗^Exp TDRD7) + (0.9419^∗^Exp TDRD5) + (−0.6324^∗^ExpPPARGC1A) + (0.9924^∗^Exp LIN28B) + (−1.0916∗Exp LRRFIP2) + (1.2895^∗^ExpPNLDC1).

First, we randomly classified the COAD patient data downloaded from the TCGA into a train group (190 patients) and a test group (189 patients), and patients of the train group were grouped into low risk, as well as the high risk on the basis of the median risk score. The results demonstrated that the OS of the high-risk and the low-risk groups were remarkably different (Figure 6(a)). Then, time-dependent ROC analysis was employed to evaluate the prognosis ability of seven-RBPs genes as shown in the figure: the AUC of the prognostic model was 0.744, which indicated moderate diagnostic performance (Figure 6(b)). After that, an expression heat map was created on basis of the 7 hub RBPs to show the risk score distribution and survival status (Figure 6(c)). Meanwhile, we analyzed the patients in the test group in the same way (Figures 7(a)–7(c)), the result of which was consistent with the previous conclusion: the AUC of the test group was 0.661, which verified the sensitivity along with the specificity of this prognostic prediction model (Figure 7(b)).

### 2.6. COX Regression Analysis of Different Clinical Parameters and Nomogram Construction

In order to study the correlation of clinical parameters with OS, we carried out univariate COX regression analyses based on key clinical characteristics. It is shown that the tumor stage, distant metastasis, primary tumor site, risk score, and regional lymph node involvement were related to OS of COAD patients (Figure 8). However, according to multiple regression analysis, age, and tumor stage along with the risk score were the only three independent prognostic variables that affect the OS (*P* value was less than or equal to 0.01) (Figure 9). Furthermore, a nomogram was constructed to set a concrete value on COAD prognosis. Specifically speaking, we obtained the total points for the one-year, three-year, and five-year survival rates according to the points corresponding to the expression of the 7 RBPs genes, so as to propose the analysis process useful for judging the prognosis of COAD to some extent (Figure 10).

## 3. Discussion

As a “transportation hub” in gene expression, RBPs regulate and participate in multiple links of posttranscriptional gene expression. This is why a series of undesirable cascading effects occur after RBPs dysregulation and eventually lead to a variety of diseases. It has been confirmed that disorder in many RBPs is linked to the onset and development of malignant tumors. To this end, we carried out a systematic analysis of COAD, a kind of malignant tumor in terms of pathology. In this study, we extracted data of COAD-related tumor tissues, as well as nontumor tissues from the TCGA data resource and screened for RBPs that were differentially expressed. Further analysis was then conducted on a biological pathway, PPI network construction, construction of prognosis-related gene model, survival time, ROC, and nomograms construction. Our goal is to have a deeper understanding of the RBPs associated with COAD and to find some biological markers with potential clinical value.

According to the GO enrichment analyses, the differently expressed RBPs were mainly involved in the following processes: modulation of translation and metabolic process, the processing and metabolic process of mRNA and ncRNA, cellular amide metabolic process, modulation of RNA splicing, RNA localization and phosphodiester bond hydrolysis, ribonucleoprotein granule, endolysosome, double-stranded RNA-binding, mRNA 3′-UTR binding, the catalytic activity acting of RNA, and ribonuclease activity. Obviously, these RBPs were demonstrated to participate in multiple biological processes such as translation, localization, binding, processing, and metabolism of RNA, which are important links for regulating posttranscriptional gene expression. Besides, RBP dysregulation will result in the occurrence along with the development of various diseases [19–21]. As a multitasking factor whose overexpression can interfere with apoptosis, cell cycle, and genome stability, the star RBP HuR is involved in multiple aspects of mRNA maturation and processing. This fact is related to the grade and malignancy of various malignant tumors including COAD [22]. IMP1 acts on mRNA related to cell growth and proliferation, thereby regulating RNA stability and affecting cell cycle progression and migration. Its overexpression is closely related to more than 80% of CRC [23]. And the overexpression of eIF4E affects the transport of specific transcripts and upregulates the translation of the GC-rich 5′-UTR mRNA sequence with a complex structure, thereby causing the occurrence and metastasis of colon cancer and other malignant tumors [24]. It is worth noting that, in our research, RBPs were remarkably abundant in the processing and metabolic process of ncRNA. At present, the analysis of RBPs is mainly based on polyadenylated mRNA-binding proteins but is merely conducted on the role of ncRNA and RBPs. It has been found that LIN28 downregulates let-7-related microRNA transcription through Lin28/let-7 axis, which eventually leads to the overexpression of multiple oncogenes (MYC, RAS, BLIMP1 [25], etc.). Nearly 30% of colorectal cancer cases are related to the above process [26, 27]. In addition, ribonucleoprotein and endosome are involved in translation and degradation, respectively. Studies have shown that heterogeneous nuclear ribonucleoprotein A1 (hnRNPA1) affects the occurrence of colorectal cancer by regulating autophagy-related gene 6 (ATG6 or Beclin-1) [28]. According to KEGG pathway analyses, the differentially expressed RBPs mainly affect the occurrence and development of colon cancer through multiple steps, such as regulating ribosome biogenesis, mRNA surveillance cascade, and RNA transport along with degradation.

After analyzing the RBPs associated with the selected key modules in the PPI network, we found that the following RBPs were mostly linked to RNA processing, splicing, metabolism, and ribonucleoprotein complex biogenesis and may result in oncogenesis. As Wnt/*β*-catenin target gene, BOP1 participated in the synthesis of the Pes1-Bop1 complex during ribosome biogenesis and promoted the metastasis of colorectal cancer cells [29, 30]. The deregulation of the BOP1 pathway increased the risk of colorectal cancer. DCAF13 has been proved to be a RAS synthetic gene in colon cancer cell lines and is related to the prognosis of liver cancer [31], breast cancer [32], and other malignant tumors. The ribosome biogenesis factor UTP14A can form a complex with ubiquitin-specific protease 36 (USP36)/Fbw7*γ*, suppress the degradation of c-Myc by Fbw7*γ*, and upregulate with c-Myc to affect colon tumor growth and metastasis [33, 34]. As a kind of RNA exosome complex, EXOSC5 participated in modulating cell proliferation, as well as the cell cycle. Studies have shown that upregulated EXOSC5 may promote the conversion of G1 phase to S phase through MAPK/ERK and PI3K/Akt signaling pathways. Meanwhile, ERK and AKT signaling stood as cyclin D1 and CDK inhibitors, which were significantly related to the size and prognosis of colorectal tumors [35]. RRP12, a conservative protein involved in ribosome biosynthesis, participates in modulating the cell cycle along with DNA damage and is associated with the occurrence of colon adenocarcinoma [36], breast cancer [37], and non-small cell lung cancer [38]. As a kind of protective gene, METTL1 participates in the modulation of cancer progression through enhancing let-7e miRNA processing in a m7G dependent-approach. It also regulated the progression of colon cancer through the METTL1/let-7e miRNA/HMGA2 cascade. Moreover, upregulation of HMGA2 was found to eliminate the inhibitory effect of METTL1 on apoptosis, invasion, and migration of colon cancer cells [39].

A prognostic model was established based on the 7 selected Hub RBPs, of which POP1, TDRD7, LRRFIP2, and PPARGC1A were identified as protective prognostic genes. Previous researches have shown that POP1, a junctional associated transmembrane protein, can inhibit the epithelial-to-mesenchymal switch. It has also been proved that POP1 is a potential tumor suppressor because of its underexpression in all stages of colorectal cancer and adenomatous polyps [40, 41]. In research on cancers, TDRD7 was sometimes taken as an interferon stimulated gene and inhibited autophagy induction [42, 43]. It is widely known that the occurrence of many tumors is closely related to autophagy dysfunction. Therefore, the biological significance of TDRD7 for malignant tumors deserves further study. In Wnt signaling pathway, LRRFIP2 can interact with Disheveled (Dvl) to increase the cellular levels of *β*-catenin and then induce lymphocyte enhancer-binding factor (LEF)/T cell factor- (TCF-) dependent transcriptional activities [44]. In addition, studies have shown that LRRFIP2 is involved in the process of alternative splicing and can affect the occurrence of colon cancer [45]. PPARGC1A participated in the regulation of mitochondrial biogenesis and energy metabolism. Interestingly, there are two diametrically opposite conclusions according to the reports of colon cancer: some studies have shown that the upregulation of PPARGC1A will increase the risk of CRC [46, 47], while others have shown that underexpression increases the risk of CRC [48, 49]. This may be due to the fact that PPARGC1A affects the occurrence of CRC through a variety of molecular mechanisms, which further illustrates that PPARGC1A is a potential favorable biological target for colorectal cancer. TDRD5, LIN28B, and PNLDC1 were identified as risky prognostic genes. TDRD5 is currently confirmed to be the piRNA biogenesis factor. And TDRD5 mRNA, whose relationship with tumors is not clear currently, is expressed in tissues of normal colon and gastric cancer [50]. Some studies have shown that TDRD5 overexpression is associated with a poor prognosis of hepatocellular carcinoma [51]. According to previous studies, PNLDC1, as a homologue of poly (A) specific ribonuclease (PARN), is likely to affect the regulation of reprogramming in early development and translation by regulating transcription products. In addition, it is found that overexpressed PNLDC1 was detected in the cytoplasm of human neoplastic spermatogenic cells. Despite the fact that the relationship between PNLDC1 and malignant tumors of the reproductive system has been revealed, more conclusive theoretical support is needed for the relationship between PNLDC1 and colon cancer [52]. LIN28B has been reviewed in the above part. In conclusion, the groups of both protective and risky prognostic genes are consistent with our grouping of models.

In summary, these screened COAD prognostic-related RBPs enjoy great prospect for research as well as a potential favorable biological target. The prognostic model we established can reflect the survival status of COAD patients. To help clinicians have a further quantitative assessment of patient survival time, we designed a nomogram for a clear reference. However, some deficiencies still exist in this experiment. First, the data used in this study are all from the TCGA database and have not been verified in other databases. Second, the database lacks clinical data to some extent, which makes our COX regression analysis of different clinical parameters not comprehensive enough. Third, more biological experiments are necessary for verifying the hub gene expression in the prognostic model although the HPA database has been utilized.

In summary, we used bioinformatics-related smart medical big data to conduct a detailed analysis of the Hub RBP with differential expression related to COAD. A COAD prognosis model was also constructed as a biological target, which can be taken as a reference for predicting COAD treatment and prognosis in future. But these results still need to be confirmed by further experimental research and clinical practice.

## 4. Materials and Methods

### 4.1. Data Sources Preprocessing

After downloading the RNA sequencing data of 398 COAD tissue samples and 39 nontumor tissue samples and their clinical data from the TCGA data resource (TCGA, https://portal.gdc.cancer.gov/), we preprocessed the original data through the Limma software package (http://www.bioconductor.org/packages/release/bioc/html/limma.html). Differentially expressed RBPs were identified based on the criteria of a false discovery rate less than 0.05 along with |log2 fold change (FC)| greater than or equal to 1. All differentially expressed RBPs with an average count value less than 1 were excluded.

### 4.2. GO and KEGG Functional Enrichment Analyses

To explore the prospective biological functions of differentially expressed RBPs, we conducted cluster enrichment analysis of these RBPs by gene ontology (GO) and the Kyoto Encyclopedia of Genes and Genomes database (KEGG) pathway, of which the GO analysis involved three components: cellular component (CC), molecular function (MF), and biological process (BP). Both P and FDR values less than 0.05 were defined as statistically significant.

### 4.3. Construction of Protein-Protein Interaction Network Pathways and Interaction Analysis

We uploaded the differentially expressed RBP data to STRING online platform (http://www.string-db.org/) to evaluate the interaction of these RBPs and then built a visual PPI network through Cytoscape 3.7.1. Through the Cytoscape Molecular Complex Detection (MCODE) plugin and with MCODE score and the node counts number more than 4 as inclusion criteria, key modules and hub genes were screened. *P* < 0.05 signified statistical significance.

### 4.4. Construction and Testing of Prognostic Model

We first conducted a univariate COX regression analysis on all differentially expressed RBPs of 190 patients' dataset from TCGA (the train group) through the survival R package and screened out candidate genes. Then, the same method was used to find hub genes based on the candidate genes, and a prognostic model was built. The risk scoring formula for each sample in the model is as follows:

Risk score = *β*1^*∗*^Exp1 + *β*2^*∗*^Exp2 + *β*_*i*_^*∗*^Exp_*i*_.

In this formula, *β* denotes the coefficient value, while Exp denotes the gene expression level. On the basis of the median risk score, we divided the patients into the high-risk group and low-risk group and conducted a log-rank test to judge the difference in OS between the two groups. In addition, the survival ROC R package was utilized to predict the sensitivity and specificity of the model. A heat map with the pheatmap package in R was made and constructed a nomogram with the R rms package to evaluate the OS. Finally, we extracted the other 189 COAD patient samples (the test group) from the TCGA database to verify the prognostic performance of the model. *P* < 0.05 represented statistical significance.

### 4.5. Validation of Expression Level

We detected the expression levels of 7 hub genes through the Human Protein Atlas (HPA) online platform (http://www.proteinatlas.org/).

## Figures and Tables

**Figure 1:** (a) Heat map and (b) volcano plot of differentially expressed RBPs in colon adenocarcinoma.

**Figure 2:** Protein interaction (PPI) network: (a) PPI network of differently expressed RBPs and Key Module, (b) Key Module 1 and (c) Key Module 2. Green circles: downregulation with a fold change of more than 4; red circles: upregulation with a fold change of more than 4.

**Figure 3:** RBPs related to the prognosis of the train group identified by univariate COX regression analysis.

**Figure 4:** RBPs related to prognosis identified by multivariate COX regression analysis.

**Figure 5:** Protein expression in normal tissues and COAD in hub genes related to prognosis verified by HPA database. (a) TDRD5. (b) LIN28B. (c) PNLDC1. (d) TDRD7. (e) LRRFIP2.

**Figure 6:** Risk score analysis of the prognostic model of COAD training group patients in the TCGA cohort. (a) Survival analysis according to risk score; (b) ROC analysis; (c) heat map and survival status.

**Figure 7:** Risk score analysis of the prognostic model of COAD test group patients in the TCGA cohort. (a) Survival analysis according to risk score; (b) ROC analysis; (c) heat map and survival status.

**Figure 8:** The prognostic value of different clinical parameters through univariate analysis (*P* < 0.01).

**Figure 9:** The prognostic value of different clinical parameters through multivariate analysis (*P* < 0.01).

**Figure 10:** Nomogram for predicting 1-, 3-, and 5-year OS of COAD patients.

**Table 1:** GO and KEGG enrichment analysis of differently expressed RBPs.

	GO term	*P* value
*Down regulated RBPs*		
Biological processes (BP)	Regulation of translation	3.22*E−*07
	Regulation of cellular amide metabolic process	9.25*E−*07
	Regulation of mRNA metabolic processing	3.42*E−*07
	Regulation of mRNA processing	1.30*E−*07
	Negative regulation of translation	2.26*E−*06
	Regulation of RNA splicing	2.48*E−*06
	Defense response to virus	1.37*E−*09
	Response to virus	2.55*E−*08

Cellular component (CC)	Endolysosome membrane	7.73*E−*06
	Endolysosome	2.39*E−*05
	Cytoplasmic ribonucleoprotein granule	0.000335342
	Ribonucleoprotein granule	0.000422761

Molecular function (MF)	mRNA 3′-UTR binding	4.75*E−*13
	mRNA 3′-UTR AU-rich region binding	2.24*E−*12
	AU-rich element binding	4.02*E−*12
	Double-stranded RNA-binding	1.52*E−*10
	Transition regulator activity	4.76*E*−07

KEGG pathway	Progesterone-mediated oocyte maturation	0.00145067
	Toll-like receptor signalling pathway	0.00167211
	Oocyte meiosis	0.00302753

*Up regulated RBPs*		
Biological processes (BP)	ncRNA metabolic process	6.50*E−*28
	ncRNA processing	2.15*E−*24
	Nucleic acid phosphodiester bond hydrolysis	1.50*E−*15
	Ribonucleoprotein complex biogenesis	3.07*E−*13
	RNA phosphodiester bond hydrolysis	7.97*E−*19
	RNA localization	3.61*E−*13
	Ribosome biogenesis	8.39*E−*15

Cellular component (CC)	Cytoplasmic ribonucleoprotein granule	3.33*E−*06
	Ribonucleoprotein granule	5.90*E−*09
	Preribosome	2.66*E−*07
	P granule	4.62*E−*06

Molecular function (MF)	Catalytic activity, acting on RNA	3.54*E−*26
	Nuclease activity	4.55*E−*14
	Ribonuclease activity	4.55*E−*14
	mRNA 3′-UTR binding	4.82*E−*10
	Catalytic activity, acting on tRNA	8.69*E−*09

KEGG pathway	Ribosome biogenesis in eukaryotes	8.34*E−*11
	RNA transport	5.55*E−*10
	mRNA surveillance pathway	1.00*E−*08
	RNA degradation	3.86*E−*05

## Data Availability

The original data utilized in this experiment are all from the TCGA website (https://portal.gdc.cancer.gov/). Here, we convey our heartfelt appreciation to the collector and producer of the research data.
